The article "Radiosensitizing Effect of Celastrol by Inhibiting G2/M Phase Arrest Induced by the c-myc Gene of Human SW1353 Chondrosarcoma Cells: Network and Experimental Analyses" was retracted in 2024. Reasons: signs of a paper mill; suspected computer-generated content; unreliable results or conclusions; concerns about the data.

# Radiosensitizing Effect of Celastrol by Inhibiting G2/M Phase Arrest Induced by the c-myc Gene of Human SW1353 Chondrosarcoma Cells: Network and Experimental Analyses

**DOI:** 10.1155/2022/1948657

**Published:** 2022-01-31

**Authors:** Jin Qian, Zhen Zhang, Xiao Han, Liulong Zhu, Zhenyu Bian, Tao Xie

**Affiliations:** Department of Orthopedic Surgery, Affiliated Hangzhou First People's Hospital, Zhejiang University School of Medicine, Hangzhou 310006, China

## Abstract

**Objective:**

Studies have unveiled that the components of *Tripterygium wilfordii* Hook F (TWHF) such as celastrol could attenuate apoptosis and proliferation of various tumor cells. This study is focused on the radiosensitization effect and apoptotic pathways of celastrol via the inhibition of the *c-myc* gene and the influence of which combined with radiotherapy on the proliferation, apoptosis, invasion, and metastasis of chondrosarcoma cells.

**Methods:**

A variety of bioinformatic tools were applied to explore the expression level and prognosis of the *c-myc* gene in different tumor cells and chondrosarcoma cells. We used pharmacology network to analyze the components, pathways, targets, molecular functions of TWHF and explore the relevant effective components over the MYC gene. Clone formation assay, CCK-8 assay, flow cytometry, and transwell migration assay were applied to detect the effects of celastrol on the expression of *c-myc* gene, cell apoptosis, and cell cycle. Radiation therapy was used to observe the radiosensitization effect of celastrol on chondrosarcoma.

**Results:**

This study shows that the c-myc gene is overexpressed in various tumor cells and bone tumor cells to varying degrees. Celastrol can significantly inhibit the expression of the *c-myc* gene, induce G2/M phase arrest through regulation of G2/M phase-related proteins, and promote SW1353 cell apoptosis through the mitochondrial signaling pathway. In addition, we also found that the use of triptorubin to inhibit *c-myc* gene expression in combination with radiotherapy can increase the osteosarcoma cells' apoptosis rate through the mitochondrial signaling pathway significantly.

**Conclusions:**

Our study validated the radiosensitization effect of celastrol through knocking down the expression of the c-myc gene to induce G2/M phase arrest and provides a new idea for the treatment of refractory or recurrent chondrosarcoma that is not sensitive to radiotherapy.

## 1. Introduction

Chondrosarcoma is a highly malignant tumor characterized by the production of the cartilage matrix by tumor cells, which is the second most commonly malignant bone tumor, with an incidence of 1 in 1,000,000 people [1, 2]. Chondrosarcoma itself has poor blood supply and lymphatic circulation and is insensitive to radiotherapy and chemotherapy; local or extensive surgical resection is the main method of treatment of chondrosarcoma to prevent local recurrence and distant metastasis [3–5]. However, for certain parts of the body, such as the pelvis or skull, it is difficult to achieve broad-side resection and the incidence of recurrence and metastasis is still high [6]. Radiotherapy is still a better palliative treatment [7, 8].

The proto-oncogene *c-myc* encodes a transcription factor c-Myc, which is of great importance in controlling cell growth and vitality. c-Myc belongs to a small family of transcription factors that contain basic, helix-loop-helix, and leucine zipper domains. c-Myc displays sequence-specific DNA-binding properties only when bound to Max, its heterodimeric partner. The interaction with Max has been shown to be necessary for most of the physiological effects of c-Myc, including the promotion of cell growth and apoptosis [9–11]. *c-myc* expression is absent in quiescent cells but is rapidly induced upon the addition of growth factors. A large body of physiological evidence shows that either upregulation or downregulation of intracellular c-Myc activity has profound consequences on cell cycle progression. There were some studies suggesting that c-Myc may stimulate the activity of cyclin E/cyclin-dependent kinase 2 (Cdk2) complexes and antagonize the action of the Cdk inhibitor p27^KIP1^. Cyclin D/Cdk4/6 complexes have also been implicated as targets of c-Myc activity. Its abnormal expression leads to 30–50% of malignant tumors, overexpression in more than 70% of human malignancies, and high expression in sarcomas [12, 13]. Overexpression of the *c-myc* gene leads to increased replication origin activity, followed by DNA damage and checkpoint activation [14, 15]. On the contrary, reducing *c-myc* expression by antisense methods or deletion of the gene by homologous recombination lead to a lengthening of the cell cycle. *c-myc* null cells display a lengthening of both the G1 and G2 phases of the cell cycle, while S phase duration remains unchanged. The expression of MYC can also induce CCNB1 to encode the mitotic driver cyclin B1, which reduces the G2/M arrest induced by DNA damage and enters inappropriate mitosis [10, 15]. Evidence showed that tumors arrest at the G2/M stage and more sensitive to radiotherapy [16]. Consequently, the combination of radiotherapy and downregulation of the c-myc gene may be a new strategy for the treatment of chondrosarcoma to deal with refractory or relapsed chondrosarcoma.

*Tripterygium wilfordii* Hook F (TWHF), a plant of the Euonymus family, has been used to treat rheumatoid arthritis as early as centuries ago and has now been used for a broad-spectrum treatment of autoimmune and inflammatory diseases [17, 18]. It contains diterpenoids such as triptolide, triterpenes such as celastrol, and other components, which have anti-inflammatory, antitumor, immunosuppressive, antioxidant, and antiobesity pharmacological effects [19, 20]. Among them, TWHF has been confirmed to be a natural proteasome inhibitor with antitumor activity [21]. With the deepening of research, it has a clear killing effect on leukemia, multiple myeloma, liver cancer, glioma, melanoma, and breast cancer [21, 22]. Related literature reports on its antitumor mechanisms are also divergent, including nuclear factor-*κ*B (nuclear factor-kappaB, (NF-*κ*B)), proteasome, mitogen-activated protein kinase (mitogen-activated protein kinase (MAPK)), and serine/threonine protein kinase B (PI3K/AKT), but it is still unclear which is its direct or main target [22–25]. At present, there is no literature report that *Tripterygium wilfordii* or some of its components can inhibit c-myc gene expression, thereby exerting antitumor effects and radiosensitization effects.

Hopkins [26] proposed the concept of network pharmacology in 2007, using bioinformatics methods to comprehensively carry out high-throughput screening and network analysis to reveal the relationship between drug components, targets, and diseases. This provides us with effective experimental assistance and theoretical basis for screening and developing drugs with high activity and low toxicity from *Tripterygium wilfordii* to treat chondrosarcoma.

In our literature, we aimed to determine the role of core components of TWHF such as celastrol in the treatment of chondrosarcoma and its potential related targets in the chondrosarcoma cell line SW1353. Meanwhile, we also attempted to observe the inhibitory effect of celastrol on the proliferation of chondrosarcoma cells and explore the mechanism of its antitumor effect. Our results demonstrated that celastrol can exert the effect of radiotherapy sensitization by inhibiting the *c-myc* gene, which provided a new method for the treatment of refractory or relapsed chondrosarcoma.

## 2. Method

### 2.1. Analysis of Pan-Cancer MYC Gene and Sarcoma Gene Expression

Gene expression matrices of different tumor and sarcoma cell lines were obtained from the Cancer Cell Line Encyclopedia (CCLE) dataset (https://portals.broadinstitute.org/ccle/about) [27], built, and visualized with R v4.0.3 package ggplot2 (v3.3.3). The limma software package (version: 3.40.2) of R software was used to study the differentially expressed mRNAs in sarcoma. The adjusted *P* value was analyzed in the Cancer Genome Atlas (TCGA) or the Genotype-Tissue Expression (GTEx) to correct false-positive results. “Adjusted *P* < 0.05 and log2 (fold change) > 1 or log2 (fold change) < −1” are defined as a threshold level for the differential expression.

### 2.2. The Prognostic Analysis of the MYC Gene for Sarcoma

The raw count of RNA sequencing data (level 3) of sarcoma and the corresponding clinical information were obtained from The Cancer Genome Atlas (TCGA) dataset (https://portal.gdc.com). The logrank was used to test the Kaplan–Meier (KM) survival analysis to compare the survival difference between the above two or more groups, and the time-dependent ROC curve (timeROC) analysis was performed to compare the prediction accuracy and risk score of the MYC gene. timeROC and the area under timeROC curve (AUC) were generated with R package “timeROC.” The *P* value and the hazard ratio (HR) with 95% confidence interval (CI) were obtained via logrank test and Cox proportional hazard regression for the Kaplan-Meier curve. All the above analysis methods and R software packages were executed using R (v4.0.3). *P* < 0.05 was considered statistically significant.

#### 2.2.1. Network Pharmacology Analysis

*(1) Search for Active Components of Tripterygium wilfordii and Related Targets*. We searched “*Tripterygium wilfordii*” in the traditional Chinese medicine systems pharmacology database and analysis platform (TCMSP) database to obtain the known pharmaceutical ingredients and all possible targets. The obtained targets were annotated through the UniProt database, and the human-derived target gene name and its ID of the corresponding target were obtained. We then searched “chondrosarcoma” in the GeneCards, OMIM, PharmGKB, TTD, DrugBank databases for related targets and aggregated and merged all potential targets for chondrosarcoma.

*(2) Construction of Protein–Protein Interactions (PPIs)*. We obtained the intersection of the drug target and disease target through R software drew the Venn diagram of the *Tripterygium*-chondrosarcoma action target to visualize the intersection of the drug-disease target. The STRING database (http://www.string-db.org) is a computerized and powerful global resource for studying the interactions between the predicted and experimental interactions of proteins. We then entered the obtained disease-drug common target set into the STRING11.0 database and set the biological category to “*Homo sapiens*,” and the interaction confidence score > 0.4, to build the PPI network. We next imported the obtained PPI network file into Cytoscape 3.8.0 software for editing and then analyzed the topological properties of the network and calculated the node's betweenness centrality (BC), closeness centrality (CC), and other related information. Genes greater than the median value were selected and saved. We finally screened twice to obtain the core target in the PPI network.

*(3) Construction of the Component-Target Network of Tripterygium wilfordii Hook F (TWHF)*. The active ingredients of TWHF and their possible targets integrated in steps 1 and 2 were regarded as two types of “nodes.” If the interaction between the drug ingredients and the target was related, “Edge” was used to connect, and Cytoscape 3.8.0 software was imported to build a “drug component-target” network. We then imported the core target obtained in step 4 into the component-target network graph, used the network analyzer to analyze the characteristic parameters of the network node, and determined the core component according to the degree.

*(4) GO and KEGG Enrichment Analyses*. Genes in modules of interest were extracted for further functional enrichment analysis. A Gene Ontology (GO) analysis was used to identify characteristic biological attributes. A Kyoto Encyclopedia of Genes and Genomes (KEGG) pathway enrichment analysis was performed to identify functional attributes. GO annotation analysis and KEGG pathway enrichment analysis of DEGs in this study were performed using the Database for Annotation, Visualization and Integrated Discovery (DAVID) tools (https://david.ncifcrf.gov/). GO was widely used to annotate functional genes, including the molecular function (MF), biological pathway (BP), and cell composition (CC). Threshold correction was set as *P* < 0.05; targets were sorted from small to large and ranked in top 10 biological processes or pathways. The top 20 pathways in the KEGG pathway were analyzed by Cytoscape to construct a “pathway-target” network. The significance of the signal pathway is indicated by the size and color of the bubble. The larger the bubble is, the more genes in the signal pathway are and the more important the pathways are.

*(5) Review and Find Target Genes and Corresponding Drug Ingredients*. We found and reviewed the active ingredients of the drug corresponding to the MYC gene and summarized the drug ingredients.

#### 2.2.2. Experimental Verification

*(1) Cell Culture and Treatment*. Cultured in DMEM containing 10% fetal bovine serum and 1% double antibody (100 U/ml penicillin and 100 *μ*g/ml streptomycin), human chondrosarcoma cells SW1353 were placed at 37°C with a 5% CO_2_ constant-temperature cell incubator. The cells in the logarithmic growth phase were digested with trypsin containing EDTA, and the chondrosarcoma cells were seeded in the cell plate and cultured for 24 hours to make them adherent. Different concentrations of TWHF were added to the treatment, and the control group was treated with 0.1% DMSO in volume fraction for 24 h and 48 h.

*(2) Cytotoxicity and Proliferation Assays*. Seeded on a 96-well plate at a density of 5 × 10^3^ cells/well, cells were incubated for 48 h in an incubator, washed twice with medium, added with 100 ml CCK-8 solution (MedChemExpress) and DMEM medium (1 : 10) mixture to each well, and incubated for 60 minutes in the dark. Minutes later, the absorbance value of each well was measured on the MR7000 microplate reader (Dynatech) at 450 nm absorbance. For cell proliferation assay, cells were cultured on 5 × 10^3^ cells/well in a 96-well plate. After drug treatment, we added CCK8 in the culture as above and measured the absorbance. According to the cell inhibition rate (%) = 1-cell survival rate, we took drug concentration as the abscissa and the cell inhibition rate as ordinate to draw the CCK-8 line chart.

*(3) Colony Formation Assay*. After the cells are treated with drugs or radiotherapy, they are seeded in a 6-well plate at 1000 cells/well and cultured at 37°C for 2 weeks. When there are macroscopic clones in the culture dish, the culture is immediately terminated. After washing 3 times with PBS, a mixture of 4% polymethanol and 0.1% crystal violet was added, fixed, and stained at 37°C for 30 minutes. Rinse the dye slowly with tap water. The count > 50 cell clones under a light microscope (magnification, ×200). Cell clone formation rate (PE) = (number of clones/number of inoculated cells) × 100%, and cell survival rate = cell clone formation rate of each experimental group/control group cell clone formation rate × 100%.

*(4) Cell Cycle Analysis*. After 0, 24, 48, 72, and 96 hours, the siRNA-transfected cells were digested and washed with PBS twice and fixed with 75% ethanol overnight in a 20°C environment. Cells were added with propidium iodide (BD Biosciences) and incubated for 15 minutes in the dark. We used the FACSCalibur flow cytometer (BD Biosciences) to analyze the cell cycle and used ModFit software to analyze the data.

*(5) Cell Apoptosis Analysis*. Annexin V FITC (Thermo Fisher) was used to analyze cell apoptosis. We digested the cells and washed them with PBS and then resuspended it in 1x binding buffer. Subsequently, we transferred the cells to 100 *μ*l of the resuspension mixture solution (1 × 10^5^ cells) into a culture tube (5 ml). V FITC (5 *μ*l) and PI (5 *μ*l) were added to the test tube and incubated at room temperature for 15 minutes. Finally, we added 400 *μ*l of 1x binding buffer to each test tube. Flow cytometry (BD Biosciences) was used for cell apoptosis analysis, and FlowJo software was used for data analysis.

*(6) Radiotherapy*. The drug-treated SW1353 cells were seeded (200 cells per well) in 6-well plates and cultured at 37°C with 5% CO_2_ for 24 hours. We used an X-ray equipment (Precision X-Ray) to irradiate cells at dose rates of 2, 4, 6, and 8 Gy. Subsequently, SW1353 cells were cultured for 10 days until colonies were visible to the naked eye.

*(7) Western Blotting*. The treated SW1353 cells were digested and lysed in RIPA lysis buffer (Sigma Aldrich). After 30 minutes, the protein concentration was measured at 570 nm wavelength by using the BCA protein analysis kit (Thermo Fisher). The same amount of protein (40 *μ*g) by SDS-PAGE (12% polyacrylamide gel) was separated.

Electrophoresis was manipulated at 100 V for 1.5 h, and the separated protein was transferred to PVDF membrane, blocked with 5% skim milk in TBS-T for 1 hour at 37°C, and incubated with primary antibody (Cell Signaling Technology) overnight at 4°C. After washing the protein three times with TBS-T, we diluted it with HRP anti-rabbit (cat. no. FD0128) or anti-mouse IgG (cat. no. FD0142) antibody (Fdbio Science) in 5% skim milk (1 : 5000) at room temperature for 1 hour. The protein bands were visualized by using WESTAR SUPERNOVA-1 Kit (Cyanagen) and Molecular Imager (Bio-Rad). We used ImageJ 1.8.0 software for density analysis.

#### 2.2.3. Data Analysis

Data were expressed as mean ± standard deviation (SD) and analyzed with SPSS17.0 (SPSS Inc.) software. We used the *t*-test to calculate the difference between the two groups and used one-way analysis of variance to compare the differences between three or more groups and then performed the Tukey post test. Two-tailed test was used for the test, and *P* < 0.05 was considered statistically significant.

## 3. Result

### 3.1. Bioinformatic Analysis of the *MYC* Gene and Chondrosarcoma Cells

We collected the *MYC* gene expression matrix of 946 different tumors and 37 sarcoma cell lines from the CCLE database, analyzed, and obtained the violin pilot of the pan-cancer analysis of the *MYC* gene (Figure 1(a)) and the difference map of the *MYC* gene expression in sarcoma cell lines, respectively (Figure 1(b)). We also made the gene expression volcano map expression (Figure 1(c)) and heat map of the differential gene expression (Figure 1(d)) of the sarcoma by acquiring the RNA sequencing data (level 3) and related information of 260 sarcomas from the TCGA database.

We then drew *MYC* gene expression and survival time and status of sarcoma patients (Figure 2(a)), as well as the distribution of the KM survival curve (Figure 2(b)), ROC curve, and AUC of the MYC gene at different times (Figure 2(c)) according to the raw count of RNA sequencing data of 260 sarcomas and corresponding clinical information from TCGA. The gene is proved to be a risk factor according to the risk score and gene expression trend after sorting gene expression from low to high (Figure 2(a)). The median overall survival (OS) of the high-expression group was 3.5 years and that of the low-expression group was 7.2 years. However, the AUC value shows that the predictive ability of the gene is general. We found that compared with normal samples, the MYC gene is overexpressed in tumor patients and sarcoma patients and MYC gene expression is in correlation negatively with the OS of patients.

### 3.2. Construction of the Compound-Target Network of *Tripterygium wilfordii* Hook F (TWHF)

We searched TCMSP (https://old.tcmsp-e.com/tcmsp.php), got 143 chemical constituents of *Tripterygium wilfordii* Hook F (TWHF) and 134 potential drug targets, and drew a CT network diagram of TWHF (Figure 3(a)), where the circles represent the active components of TWHF and the squares represent the drug targets. It shows that multiple active ingredients act on multiple targets, reflecting the multicomponent and multitarget synergistic treatment characteristics of TWHF. We collected 802, 4, 1714, 0, and 0 potential chondrosarcoma targets from GeneCards, OMIM, PharmGKB, TTD, and DrugBank, respectively. We summarized and merged all data and obtained a total of 2419 chondrosarcoma-related targets (Figure 3(b)).

### 3.3. Construction of Protein–Protein Interactions (PPIs)

After summarizing the previously-obtained drug and disease targets, we obtained 104 active ingredient-disease common targets by using the R language to take the intersection and draw the Venn diagram (Figure 3(c)). STRING 11.0 was applied to analyze common targets and collect protein interactions. In STRING, the confidence score was set more than 0.4 and the isolated edges was deleted. The PPI network has 104 nodes and 1631 edges and the average degree of this network is 31.4 (Figure 4). We then used Cytoscape 3.8.0 software to revisualize and analyze the active ingredient-disease common target network. The larger the node and the darker the color is, the higher the degree parameter value is, indicating that it may be the key target to find. After filtering the nodes twice according to each parameter, 18 nodes and 153 edges are finally obtained (Figure 4). It is confirmed that the core targets obtained in the final screening are MAPK8, VEGFA, CASP3, CXCL8, TP53, FOS, MMP9, IL6, AKT1, TNF, JUN, STAT3, MAPK14, PTGS2, MYC, MMP2, MAPK1, and RELA.

### 3.4. GO and KEGG Enrichment Analyses

GO enrichment analysis was used, and we obtained 1908 items related to biological processes, 35 items related to cell components, and 145 items related to molecular functions, which were sorted and summarized according to the corrected *P* value (Table 1) and plotted as a histogram (Figure 5(a)). We got 144 items through KEGG pathway analysis, and the top 30 items were screened out based on the corrected *P* value, and a bubble chart (Figure 5(b) and Table 2) and a cell cycle pathway diagram were drawn (Figure 5(c)).

### 3.5. Analysis of *MYC* Gene-Targeted Drugs

Having reviewed the information collected in network pharmacology, we found that celastrol (NSC 70931) is the only drug component of TWHF that targets the *MY*C gene. We then analyzed and summarized the corresponding targets of celastrol (Table 3).

### 3.6. Celastrol Inhibits SW1353 Proliferation and Induces Caspase-Dependent Cell Apoptosis

We first investigated the influence of celastrol (0, 1.0, 2.0, 3.0, 4.0, and 5.0 *μ*M) on human chondrosarcoma cells SW1353. The cell proliferation assay (Figure 6(a)) and the clone formation assay (Figure 6(b)) showed that celastrol not only inhibits the cell viability of the SW1353 cell lines in a dose-dependent manner but also in a time-dependent manner. The maximum inhibition rate of celastrol appeared at 48 hours at 5.0 *μ*M (Figure 6(a)).

The apoptosis assay (Figure 6(c)) showed that the proportion of early and late apoptotic cells in SW1353 increased after celastrol treatment. The involved pathways were determined by Western blotting (Figure 6(d)). Celastrol inhibits the expression of the *c-myc* gene, increases the expression of cleaved PARP and cleaved caspase-3 protein, and reduces caspase-9, caspase-3, Bid, Bcl-2, Bax, and PARP protein expression. The ratio of Bcl-2/Bax was reduced by gray analysis. Above that, the apoptosis caused by *Tripterygium wilfordii* may be related to the mitochondrial signaling pathway.

The results of cell cycle detection by flow cytometry (Figure 7(a)) showed that the proportion of cells in the G2 phase in the control group and the 0.5, 1.0, and 1.5 *μ*M triptoerygrin intervention groups were 14.07%, 25.79%, 24.07%, and 22.45%, respectively, which indicate that the drug can block the cell cycle of chondrosarcoma at the G2/M stage and is concentration dependent. When the concentration of TWHF reaches 1 *μ*M (about half of the IC50), the maximum arrest in the G2/M stage occurs accompanied by an increase in the proportion of the S phase. Western blotting assay showed that the expression of cell cycle regulatory proteins p21, cyclin D1, cyclin B1, and Cdc2 was downregulated (Figure 7(b)), which may be the direct cause of G2/M phase arrest.

### 3.7. Measure the Radiosensitivity of SW1353 Cells

SW1353 cells were irradiated with 2, 4, 6, and 8 Gy to determine their radiosensitivity. As shown in Figure 7(c), the colony survival rates calculated based on the number of communities in the radiotherapy group/the number of communities in the NC group were 71.3%, 29.3%, 58%, and 0.0%, respectively. The cell survival rate was significantly reduced in a dose-dependent manner. In order to rule out that the intensity of radiotherapy directly leads to cell death, the radiation dose of 2 Gy is used in subsequent radio sensitization experiments.

### 3.8. Celastrol Achieves the Effect of Radiotherapy Sensitization by Inducing G2/M Phase Arrest

According to the clone formation experiment (Figure 8(a)), the average number of colonies in the NC, celastrol, 2 Gy, and celastrol + 2 Gy groups with a seeding density of 200/well were 81, 54, 51, and 9, respectively, and the colony formation rate in the celastrol + 2 Gy group is significantly reduced. Western blot analysis showed (Figure 8(b)) that the expression of cell cycle regulatory proteins cyclinB1 and p21, Cdc2, and cyclinD1 in the celastrol and celastrol + 2 Gy groups was downregulated. Apoptosis-related proteins c-myc, caspase-9, caspase-3, Bid, Bcl-2, Bax, and PARP protein expression decreased, while cleaved PARP and cleaved caspase-3 protein expression increased. The result confirms that the combination therapy promotes the apoptosis of chondrosarcoma, which is attributed to the radiosensitization effect of celastrol by downregulating the expression of c-myc and inducing the G2/M phase arrest and the induction of chondrosarcoma apoptosis through the mitochondrial signaling pathway.

## 4. Discussion

Chondrosarcoma was strongly resistant to X-rays, which has caused great limitations in the treatment of chondrosarcoma [7]. Accumulating evidence indicates that cell cycle G2/M phase arrest is one of the key factors to enhance the sensitivity of radiotherapy [15, 28, 29]. Inhibition of *c-myc* expression can effectively inhibit tumor cell proliferation and induce G2/M phase arrest and apoptosis of sarcoma cells [15, 30–33]. This study shows that celastrol can effectively inhibit the expression of the *c-myc* gene and significantly inhibit the growth of tumors. At the same time, celastrol can promote the radiosensitization caused by G2/M phase arrest by inhibiting the expression of the c-myc gene and enhance the apoptosis caused by the mitochondrial signaling pathway.

Through bioinformatics analysis, we found that the *MYC* gene is highly expressed in a variety of tumor and sarcoma cell lines to varying degrees and is negatively correlated with the OS of patients. Many components of TWHF have been confirmed to have antitumor activity, but no reports have been found on drug components directly related to the MYC gene [34, 35]. Through the network pharmacology summary, we revealed that *Tripterygium wilfordii* has the characteristics of multicomponent, multipathway, multitarget, multibiological function, etc., playing a therapeutic effect on chondrosarcoma, and found its biological process in GO enrichment analysis (BP is related to response to radiation, CC is related to cyclin-dependent protein kinase, and MF is related to transcription factor binding). This laid the foundation for us to find a good radiosensitizer and *MYC* gene inhibitor in the active ingredients of TWHF. The proto-oncogene *c-myc* encodes a transcription factor c-Myc, which is greatly important in controlling cell growth and vitality. The quantity of c-Myc is carefully controlled by many mechanisms, and its actions to induce and repress genes are modulated by interactions with other regulatory proteins. Previous studies showed that celastrol inhibits chondrosarcoma proliferation, migration, and invasion through suppression of the CIP2A/c-MYC signaling pathway. We discovered that celastrol was the only active component of the drug related to the *MYC* gene, and its drug targets are mostly related to radiation, which is consistent with the literature report [36].

Radiotherapy has become an important part of cancer treatment [37]. Radiation therapy induces apoptosis by destroying DNA and inhibiting checkpoint activation of the cell cycle [38, 39]. As a response to DNA damage, cells mainly stagnate at the junction of cell checkpoints G1/S and G2/M, which is the core mechanism that controls DNA replication and repair and cell division in eukaryotic cells [15]. G1/S arrest prevents damaged DNA from entering the S phase, and G2/M arrest prevents damaged DNA from entering mitosis. Therefore, in order to deal with DNA damage, normal cells prevent the activation of Cdc2/cyclin B through various mechanisms, such as the cytoplasmic isolation of the key components of Cdc2 activation (cyclin B and Cdc25C) [10, 15]. Therefore, how to reduce the cyclin B1/Cdc2 complex and induce cell G2/M arrest is the key to sensitizing tumor cells to the effect of radiotherapy.

Tumor cells have a strong ability to proliferate and are accompanied by cell cycle disorders. The *c-myc* gene can directly induce the high expression of the cell cycle-regulating genes CDC2-L1 and Cyclin B1 and can maintain the abnormally high expression of cyclin B1 under the induction of ionizing radiation (IR), causing the cells with DNA damage to enter inappropriately the S phase, thereby enhancing the resistance to ionizing radiation [15, 30, 40].

In *in vitro* experiments, we found that celastrol can effectively inhibit the expression of the *c-myc* gene and reduce the expression of cyclin B1 and Cdc2 (CDK1) proteins, resulting in chondrosarcoma cell G2/M phase arrest and effective inhibition proliferation of chondrosarcoma cells [29, 41]. Although c-Myc gene is related to caspase-3 related pathways to promote cell apoptosis, inhibiting the cyclin B1/Cdc2 complex and inducing G2/M phase arrest are still the main driving forces for inhibiting the c-myc gene to control tumorigenesis [11, 16, 28]. We also found that the expression of P21 protein in chondrosarcoma cells decreased with the increase of drug concentration, which may be related to the multitarget effect of celastrol and the time of action of drugs or radiation. Further research is needed [5, 7, 42]. In vitro experiments confirmed that celastrol can interfere with cyclin-dependent protein kinases by inhibiting the *MYC* gene-encoding transcription factors and lead to radiosensitization, which verified the accuracy of the conclusions of network pharmacology.

In summary, this study proved that celastrol can inhibit the proliferation of chondrosarcoma cells by downregulating the *c-myc* gene and induce cell cycle arrest in the G2/M phase. At the same time, the combined application of radiotherapy and celastrol makes the apoptosis rate of chondrosarcoma cells significantly higher than that of any single treatment method. This method can not only reduce the liver and kidney toxicity caused by the single use of large doses of drugs but also reduce the impact of the single use of large doses of radiotherapy on the cells of the whole body. Therefore, we believe that celastrol is a radiosensitizer that inhibits the expression of the *c-myc* gene and is an effective strategy to improve the sensitivity of clinical tumor radiotherapy, providing a new way of treatment for chondrosarcoma.

## Figures and Tables

**Figure 1:** The differential expression of the myc gene and the differential analysis of sarcoma cell lines. (a) The expression distribution of the MYC gene in different tumor tissues. (b) The expression distribution of the MYC gene in sarcoma cell lines. (c) Volcano plots. (d) Hierarchical clustering analysis of mRNAs.

**Figure 2:** Prognostic analysis of the gene signature in the TCGA set. (a) TCGA dataset. (b) KM survival curve distribution of the MYC gene in the TCGA dataset. (c) ROC curve and AUC of the gene at different times.

**Figure 3:** Construction of the C-T network of TWHF for chondrosarcoma treatment. (a) Constructing the relationship between all the therapeutic targets of TWHF and all the drug components. (b) The intersection of chondrosarcoma target genes in different databases. (c) The intersection of TWHF treatment targets and chondrosarcoma disease targets. (d) Constructing a PPI network of TWHF for the treatment of chondrosarcoma based on STRING.

**Figure 4:** Obtaining the core target of TWHF for the treatment of chondrosarcoma.

**Figure 5:** Gene enrichment analysis based on GO and KEGG. (a) Histogram of GO function enrichment at the intersection target of TWHF and chondrosarcoma. (b) Histogram of KEGG enrichment at the intersection target of TWHF and chondrosarcoma. (c) Schematic diagram of core genes involved in the cell cycle pathway enrichment based on KEGG analysis.

**Figure 6:** TWHF inhibits the proliferation of osteosarcoma cells by inhibiting the expression of the C-myc gene and induces caspase-dependent cell apoptosis. (a) Cell survival rate and drug IC50. (b) Colony formation assay. (c) Flow cytometry assay. (d) Western blotting detects the caspase-dependent apoptosis pathway.

**Figure 7:** Celastrol influences the cell cycle of SW1353 by regulating cell cycle regulator proteins and assesses its radiosensitivity. (a) Flow cytometry analysis. (b) Western blotting. (c) SW1353 cells were irradiated with 0, 2, 4, 6, and 8 Gy, colony formation experiments were performed, and the radiosensitivity of the cells was evaluated.

**Figure 8:** Celastrol downregulates the c-myc gene and induces G2/M phase block to cause radiosensitization of SW1353 cells. (a) The radiosensitization caused by celastrol was detected by the colony formation experiment. (b) Western blotting proved that the radiosensitization effect caused by t celastrol is to induce SW1353 cell apoptosis through the regulation of cycle regulator proteins and through the mitochondrial signaling pathway.

**Table 1:** Summary of GO function enrichment of *Tripterygium wilfordii* Hook F (TWHF) chondrosarcoma targets.

Ontology	ID	Description	*P*.adjust
BP	GO:0032496	Response to lipopolysaccharide	2.00*E* − 22
	GO:0002237	Response to molecule of bacterial origin	5.25*E* − 22
	GO:0042493	Response to drug	9.74*E* − 22
	GO:0070482	Response to oxygen levels	4.77*E* − 16
	GO:0048545	Response to steroid hormone	5.18*E* − 14
	GO:0009411	Response to UV	5.26*E* − 14
	GO:0097191	Extrinsic apoptotic signaling pathway	7.06*E* − 14
	GO:0051090	Regulation of DNA-binding transcription factor activity	8.31*E* − 14
	GO:0009314	Response to radiation	8.55*E* − 14
	GO:2001237	Negative regulation of extrinsic apoptotic signaling pathway	1.35*E* − 13

CC	GO:0005759	Mitochondrial matrix	1.07*E* − 07
	GO:0045121	Membrane raft	1.15*E* − 06
	GO:0098857	Membrane microdomain	1.15*E* − 06
	GO:0005667	Transcription regulator complex	1.03*E* − 05
	GO:0031968	Organelle outer membrane	1.03*E* − 05
	GO:0019867	Outer membrane	1.03*E* − 05
	GO:0005741	Mitochondrial outer membrane	2.93*E* − 05
	GO:0000307	Cyclin-dependent protein kinase holoenzyme complex	8.19*E* − 05
	GO:0090575	RNA polymerase II transcription regulator complex	8.19*E* − 05
	GO:1904813	Ficolin-1-rich granule lumen	9.39*E* − 05

MF	GO:0140297	DNA-binding transcription factor binding	1.17*E* − 09
	GO:0061629	RNA polymerase II-specific DNA-binding transcription factor binding	6.55*E* − 08
	GO:0033613	Activating transcription factor binding	6.55*E* − 08
	GO:0001216	DNA-binding transcription activator activity	2.30*E* − 06
	GO:0031072	Heat shock protein binding	2.30*E* − 06
	GO:0005126	Cytokine receptor binding	2.41*E* − 06
	GO:0002020	Protease binding	2.85*E* − 06
	GO:0005125	Cytokine activity	4.09*E* − 06
	GO:0005178	Integrin binding	4.45*E* − 06
	GO:0001228	DNA-binding transcription activator activity, RNA polymerase II specific	6.10*E* − 06

**Table 2:** Summary table of KEGG function enrichment of TWHF-chondrosarcoma targets.

ID	Description	*P*.adjust
hsa05417	Lipid and atherosclerosis	8.28*E* − 27
hsa05163	Human cytomegalovirus infection	4.15*E* − 25
hsa05167	Kaposi sarcoma-associated herpesvirus infection	1.62*E* − 23
hsa04933	AGE-RAGE signaling pathway in diabetic complications	2.37*E* − 23
hsa05161	Hepatitis B	2.37*E* − 23
hsa04668	TNF signaling pathway	8.76*E* − 21
hsa05418	Fluid shear stress and atherosclerosis	6.58*E* − 20
hsa04657	IL-17 signaling pathway	8.02*E* − 20
hsa05166	Human T-cell leukemia virus 1 infection	1.12*E* − 18
hsa04210	Apoptosis	1.16*E* − 17
hsa05222	Small cell lung cancer	2.72*E* − 17
hsa05160	Hepatitis C	2.41*E* − 16
hsa05162	Measles	2.71*E* − 16
hsa05169	Epstein-Barr virus infection	2.86*E* − 16
hsa05145	Toxoplasmosis	1.01*E* − 15
hsa05215	Prostate cancer	1.26*E* − 15
hsa01522	Endocrine resistance	1.43*E* − 15
hsa05142	Chagas disease	2.87*E* − 15
hsa04151	PI3K-Akt signaling pathway	1.42*E* − 14
hsa05205	Proteoglycans in cancer	4.71*E* − 14
hsa05212	Pancreatic cancer	1.64*E* − 13
hsa04926	Relaxin signaling pathway	1.75*E* − 13
hsa05219	Bladder cancer	4.46*E* − 13
hsa04915	Estrogen signaling pathway	5.38*E* − 13
hsa05170	Human immunodeficiency virus 1 infection	8.36*E* − 13
hsa05207	Chemical carcinogenesis-receptor activation	8.36*E* − 13
hsa05224	Breast cancer	1.47*E* − 12
hsa04932	Nonalcoholic fatty liver disease	3.60*E* − 12
hsa05152	Tuberculosis	4.16*E* − 12
hsa04064	NF-kappa B signaling pathway	1.41*E* − 11
hsa04620	Toll-like receptor signaling pathway	1.41*E* − 11

**Table 3:** Summary of celastrol information.

Drug name	Target	Symbol
*Tripterine*	NR3C1	Glucocorticoid receptor
	VEGFA	Vascular endothelial growth factor A

MOL003186	CCND1	G1/S-specific cyclin-D1
	BCL2	Apoptosis regulator Bcl-2
	BCL2L1	Bcl-2-like protein 1

	BAX	Apoptosis regulator BAX
	FLT1	Vascular endothelial growth factor receptor 1
	KDR	Vascular endothelial growth factor receptor 2
	MMP9	Matrix metalloproteinase-9
	JUN	Transcription factor AP-1
	PTGS2	Prostaglandin G/H synthase 2
	BIRC5	Baculoviral IAP repeat-containing protein 5
	BIRC2	Baculoviral IAP repeat-containing protein 2
	CFLAR	CASP8 and FADD-like apoptosis regulator
	AKR1B1	Aldose reductase
	CDC37	Hsp90 cochaperone Cdc37
	MMP2	72 kDa type IV collagenase
	TIMP1	Metalloproteinase inhibitor 1
	TIMP2	Metalloproteinase inhibitor 2
	MMP1	Interstitial collagenase
	**MYC**	Myc proto-oncogene protein
	FNDC3B	Fibronectin
	COL7A1	Collagen alpha-1 (VII) chain
	COL4A4	Transforming growth factor beta-1
	RELA	Collagen alpha-4 (IV) chain

## Data Availability

The authors confirm that the data supporting the findings of this study are available within the article.
